The article "Study on the Effects of Chinese Materia Medica Processing on the Hypoglycemic Activity and Chemical Composition of Anemarrhenae Rhizoma" was published in 2021. Journal: Evid Based Complement Alternat Med.

# Study on the Effects of Chinese Materia Medica Processing on the Hypoglycemic Activity and Chemical Composition of Anemarrhenae Rhizoma

**DOI:** 10.1155/2021/6211609

**Published:** 2021-10-19

**Authors:** Ying-Qi Yu, Li Yan, Xiao-Ting Wang, Li Li, Wei Zheng, Hui Gao

**Affiliations:** College of Pharmacy, Liaoning University of Traditional Chinese Medicine, Shenyang, China

## Abstract

**Purpose:**

To compare the hypoglycemic effects of different extracts of Anemarrhenae Rhizoma (AR) before and after being stir-baked with salt water on the diabetic mice and to detect the contents of 8 components in the corresponding active parts simultaneously using the UPLC-MS method, in order to screen the better extracts for diabetes and to clear the material basis for enhancing hypoglycemic activity of Anemarrhenae Rhizoma stir-baked with salt water (SAR).

**Methods:**

Taking spontaneous type II diabetic db/db mice as models and fasting blood glucose (FBG), oral glucose tolerance test (OGTT), glycated hemoglobin or glycosylated hemoglobin (HbAlc), serum resistin (RESISTEIN), fasting insulin (FINS), superoxide dismutase (SOD), malondialdehyde (MDA), and nitric oxide (NO) as indicators, the hypoglycemic effects of different active parts of Anemarrhenae Rhizoma were evaluated. The chromatographic separation was performed on a Waters BEH C18 (2.1 mm × 50 mm, 1.7 *μ*m) column using acetonitrile (B) and 0.1% formic acid in water (*A*) as mobile phases, and the flow rate was 0.3 ml/min. The column temperature was set as 28°C, and the injection volume was 10 *μ*L. A mass spectrometer was connected to the UPLC system via an electrospray ionization (ESI) interface. Full-scan data acquisition was performed in the negative ion mode.

**Result:**

In the study of pharmacodynamics, the hypoglycemic effect of Anemarrhenae Rhizoma stir-baked with salt water is better than that of Anemarrhenae Rhizoma and the hypoglycemic effect of ethanol extract of Anemarrhenae Rhizoma is more remarkable than that of the decoction. The measured components all have a good linear relationship within their respective linear ranges (*r* ≥ 0.9990); the average recovery rates are 98.86%–100.69%, RSD <2.90%. Compared with the raw Anemarrhenae Rhizoma, the contents of Timosaponin AIII, Timosaponin BII, Timosaponin BIII, Anemarrhenasaponin I, Anemarrhenasaponin Ia, and Mangiferin of Anemarrhenae Rhizoma stir-baked with salt water are all higher, the changes of Timosaponin AI and Anemarrhenasaponin AII are not obvious, and all the contents of chemical composition in the ethanol extract of Anemarrhenae Rhizoma and Anemarrhenae Rhizoma stir-baked with salt water were obviously higher compared with the water decoction.

The article "Study on the Effects of Chinese Materia Medica Processing on the Hypoglycemic Activity and Chemical Composition of Anemarrhenae Rhizoma" was published in 2021. Journal: Evid Based Complement Alternat Med.

**Conclusion:**

The processing method, stir-baking with salt water, can increase the contents of active compositions in Anemarrhenae Rhizoma and strengthen the hypoglycemic effect. The ethanol extract of Anemarrhenae Rhizoma stir-baked with salt water is the better active site.

## 1. Introduction

Traditional Chinese medicine (TCM) has its unique theoretical system and application form. Chinese material medica processing can reduce the toxicity of TCM and increase its efficiency, which is an indispensable guarantee for effectiveness and safety of traditional Chinese medicine clinical practice [1]. TCM processing is a unique and traditional pharmaceutical technology adopted according to the theory of TCM, the nature of Chinese crude drug, and the needs of dispensing preparation and clinical application. TCM processing makes TCM different from natural medicine [2]. TCM processing was listed in the first batch of national intangible cultural heritage in 2006. TCM processing is a major feature on the clinical prescription of TCM. Raw decoction pieces and processed decoction pieces are used for different symptoms. There are many records in ancient books to guide Chinese medicine practitioners to use processed products; meantime, the researchers of traditional Chinese medicine processing have been struggling to explain different treatments of raw and cooked by analyzing the changes of pharmacodynamic substances and the regular pattern of the body's action caused by the processing of TCM [3].

Anemarrhenae Rhizoma refers to the dry rhizome of the plant *Anemarrhena asphodeloides* Bge. of the family Liliaceae. It is bitter and sweet with cold nature and attributive to lung, stomach, and kidney meridians, taking on effects of heat-clearing, fire-purging, nourishing Yin, and moisturizing dryness [4]. In clinical Chinese medicine, in addition to the use of AR, there is also the application of SAR, which has a history of nearly a thousand years. The traditional theory of TCM believes that the processing method, stir-baking with salt water, can introduce the medicines into the kidney meridian and enhance the effect of nourishing Yin for lowering fire. Our research has found that the stir-baking with salt water can enhance the hypoglycemic effect of Anemarrhenae Rhizoma (AR) significantly, which is just consistent with the traditional theory of the processing of AR because TCM believes that the main pathogenesis of diabetes is the loss of Yin and Jin and the excessive dryness and heat. The deficiency of Yin is the root cause, and the dryness and heat are the superficies [5]. Anemarrhenae Rhizoma stir-baked with salt water (SAR) can improve this symptom properly. In order to explain the processing effect of AR from the chemical composition and medicinal effect, domestic researchers of traditional Chinese medicine have done a lot of research on the hypoglycemic effect of traditional Chinese medicine [6], but there are few studies on the synergistic effect of hypoglycemic effect after processing. In order to explain the processing principle of the hypoglycemic effect of SAR, we have carried out many experimental studies. The research studies on the hypoglycemic effect of SAR have been reported mainly by our research group until now. We found the contents of three components, Timosaponin AIII, Timosaponin BIII, and Mangiferin, increased in the SAR and confirmed the hypoglycemic activity of these three components [7].

The article "Study on the Effects of Chinese Materia Medica Processing on the Hypoglycemic Activity and Chemical Composition of Anemarrhenae Rhizoma" was published in 2021. Journal: Evid Based Complement Alternat Med.

On the basis of previous research, this thesis used spontaneous type 2 diabetic db/db mice as experimental animals and used fasting blood glucose (FBG), oral glucose tolerance test (OGTT), glycated hemoglobin or glycosylated hemoglobin (HbAlc), serum resistin (RESISTEIN), fasting insulin (FINS), superoxide dismutase (SOD), malondialdehyde (MDA), and nitric oxide (NO) as indicators to evaluate the hypoglycemic effects of water decoction from AR (WAR) and SAR (WSAR) and ethanol extract from AR (EAR) and SAR (ESAR), and ultraperformance liquid chromatography coupled with a triple quadrupole mass spectrometry (UPLC-QQQ-MS/MS) was used to analyze the changes in the contents of Timosaponin AIII, Timosaponin BII, Timosaponin BIII, Mangiferin, Anemarrhenasaponin I, Anemarrhenasaponin Ia, Timosaponin AI, and Anemarrhenasaponin AII before and after being stir-baked with salt water. Combining the results of the efficacy and the component analysis, the principle of Chinese materia medica processing can be illustrated, that is, to explain why the hypoglycemic effect of SAR can be enhanced.

## 2. Instruments and Materials

### 2.1. Instruments

The instruments used were as follows: Waters Xevo TQD triple four-stage rod liquid chromatography (Waters Company, United States), one-hundredth analytical balance (METTLER AE240, Switzerland), electronic balance (FA10004 B, Shanghai Precision Scientific Instrument Co., Ltd.), Whirlpool Mixer (Shanghai Qingpu Huxi Instrument Factory), horizontal ultralow temperature preservation box (Qingdao Haier Special Electrical Appliances Co., Ltd.), 250 g swing high-speed universal crusher (Wenling Jida Machinery Co., Ltd.), Integrated Milli-Q Integral (Milli Co., Ltd.), CNC ultrasonic cleaner (KQ-250DB, Kunshan Ultrasound Instrument Co., Ltd.), electric thermostat water bath pot (Beijing), Multiskan MK3 enzyme labeling instrument (Semefield Technology Co., Ltd.), TGL-16C table centrifuge (Shanghai Anting Scientific Instrument Factory), blood glucose instrument (Bayer Medical and Health Co., Ltd.), rotary evaporator (Shanghai Yarong Biochemical Instrument Factory), PH acidimeter (Shanghai Peng Science Co., Ltd.), and MassLynx V4.1.

The article "Study on the Effects of Chinese Materia Medica Processing on the Hypoglycemic Activity and Chemical Composition of Anemarrhenae Rhizoma" was published in 2021. Journal: Evid Based Complement Alternat Med.

### 2.2. Materials

Timosaponin AI (purity ≥98%, no. MUST-17022810), Anemarrhenasaponin AII (purity ≥98%, no. MUST-16112415), Timosaponin BII (purity ≥98%, no. MUST-17040602), Timosaponin BIII (purity ≥98%, no. MUST-1702210), Anemarrhenasaponin I (purity ≥98%, no. MUST-16112412), and Anemarrhenasaponin Ia (purity ≥98, no. MUST-16112413) were all purchased from Chengdu Biotechnology Co., Ltd.; Mangiferin (purity ≥98%, no. 160101), Sichuan Vicki Biotechnology Co., Ltd.; Timosaponin AIII (purity ≥98%, homemade). Blood glucose test paper (Bayer Medical and Health Co., Ltd.); HbAlc reagent kit (lot no. 20170512DB); mouse serum insulin (INS) reagent kit (lot no. 20170415BE); mouse serum resistin (RESISTIN) reagent box (lot no. 20170412MU); mouse nitric oxide (NO) kit (lot no. 20170411YS); mouse superoxide dismutase (SOD) kit (lot no. 20170411XE); mouse malondialdehyde (MDA) kit box (Shanghai Langdon Biotechnology Co., Ltd., lot no. 20170409CS). Anemarrhenae Rhizoma (Sichuan New Lotus Chinese Medicine Decoction Co., Ltd., batch no. 1510038) was identified as the dried rhizome of *Anemarrhena asphodeloides* Bge. by Professor Yanjun Zhai of Liaoning Traditional Chinese Medicine University.

### 2.3. Animals

There were 30 healthy SPF 7–9-week-old male db/db mice and 6 db/m mice, weighing 50 g–60 g, provided by Changzhou Card Vince Laboratory Animal Co., Ltd. All experiments involving animals were approved by the Animal Care and Welfare Committee of Liaoning University of Traditional Chinese Medicine (use license no. SYXK(Liao)2019–0004).

## 3. Experimental Method

### 3.1. Effects of Anemarrhenae Rhizoma on Hypoglycemic Activity in db/db Mice

#### 3.1.1. Sample Preparation

Add 30 mL salt water (containing 3 g salt) to every 100 g AR decoction pieces, mix well and stir thoroughly, and stir-bake at 150°C∼160°C for 8 min [8].

Preparation of water decoction: weigh AR/SAR decoction pieces, add 15 times the amount of water to a group and decoct 3 times, each time for 1 h, filter the combined water decoction, and concentrate to make the concentration of 0.25 g·mL^−1^ of AR and SAR water decoction, respectively.

Preparation of ethanol extract: AR/SAR was extracted 3 times with 15 times the amount of 75% ethanol under reflux, 1 h each time, filtered, combined the filtrate, and concentrated until no alcohol smell to obtain the extract, which was dispersed in water to prepare ethanol extract of AR and SAR with a concentration of 0.25 g·mL^−1^, respectively.

The article "Study on the Effects of Chinese Materia Medica Processing on the Hypoglycemic Activity and Chemical Composition of Anemarrhenae Rhizoma" was published in 2021. Journal: Evid Based Complement Alternat Med.

#### 3.1.2. Grouping and Administration

After adaptive feeding for 7 days and fasting for 12 hours, blood was collected from the tail vein to determine the fasting blood glucose level. The mice whose average blood glucose level was ≥11.0 mmol L^−1^ [9] can be used for experiments. Number the db/db mice with qualified blood glucose, and randomly group them using the Syntax window in SPSS. Numbers 1–6 are the db/db control group, numbers 7–12 and 13–18 are the raw and salt Anemarrhenae water decoction groups, respectively, and numbers 19–24 and 25–30 are the raw and salt Anemarrhenae ethanol extract groups, respectively; db/m is the normal control group. Except for the db/m normal control group and the db/db control group, each group was given the corresponding liquid medicine for 2 weeks (5 g kg^−1^ d^−1^).

#### 3.1.3. The Effect on Fasting Blood Glucose (FBG) [10] in Spontaneous Type 2 Diabetic db/db Mice

After 7 days and 14 days of administration and fasting for 12 hours, blood was collected from the tail vein, and a blood glucose meter was used to determine the fasting blood glucose of mice (FBG).

#### 3.1.4. The Effect of Glucose Tolerance (OGTT) [11] in Spontaneous Type 2 Diabetic db/db Mice

After the last blood glucose measurement, a glucose solution (2 g·kg^−1^) was administered by gavage. The blood glucose value and the area under the curve (AUC) were measured for 0 h, 0.5 h, 1 h, and 2 h, and the glucose tolerance (OGTT) was calculated.

#### 3.1.5. The Effects of HbAlc, RESISTEIN, FINS, SOD, MDA, and NO in Type 2 Diabetic db/db Mice

After the last dose and fasting for 12 hours, take blood from the mouse abdominal aorta, centrifuge, and take serum and plasma; then, take pancreatic tissue, homogenize, and determine glycosylated hemoglobin (HbAlc) [12], serum resistin (RESISTEIN) [13], and serum insulin (FINS) [14] according to the instructions of the enzyme linked immunosorbent assay (ELISA) kit, and calculate the islet sensitivity index (ISI) and insulin resistance index (HOMA-IR) according to the following formulas: ISI = ln[1/(FBG × FINS)]; HOMA-IR = FBG × FINS/22.5 [15]. Then, determine superoxide dismutase (SOD) [16], malondialdehyde (MDA) [17], and nitric oxide (NO) [18] in pancreatic tissue content.

### 3.2. The Influence of Processing on the Compounds in Anemarrhenae Rhizoma

#### 3.2.1. Preparation of Sample Solution

Weigh raw and salt *Anemarrhena* powder separately (each 10 g), and prepare the extract as described in Section 3.1.1 and then weigh, dissolve with 100 ml methanol, filter, and pass through a 0.22 *μ*m microporous filter membrane. Take additional filtrate and set aside.

The article "Study on the Effects of Chinese Materia Medica Processing on the Hypoglycemic Activity and Chemical Composition of Anemarrhenae Rhizoma" was published in 2021. Journal: Evid Based Complement Alternat Med.

#### 3.2.2. Preparation of Reference Solution

Precisely weigh the Timosaponin AI, Timosaponin AIII, Timosaponin BII, Timosaponin BIII, Anemarrhenasaponin I, Anemarrhenasaponin Ia, Anemarrhenasaponin AII, and Mangiferin reference substances, put in a 10 mL volumetric flask, and add methanol to dilute to the mark. The concentrations are, respectively, Timosaponin AI (1.10 g·mL^−1^), Anemarrhenasaponin AII (1.04 g·mL^−1^), Timosaponin AIII (1.14 g·mL^−1^), Timosaponin BII (1.06 g·mL^−1^), Timosaponin BIII (1.48 g·mL^−1^), Anemarrhenasaponin I (1.03 g·mL^−1^), Anemarrhenasaponin Ia (1.21 g·mL^−1^), and Mangiferin (1.63 g·mL^−1^), stored in a refrigerator at 4°C. Dilute with methanol and water before use to obtain mixed reference substance stock solutions of different mass concentrations. It is used for the determination of linear investigation and content determination.

#### 3.2.3. Chromatographic Conditions

A Waters BEH C18 column (2.1 mm × 5 0 mm, 1.7 *μ*m) is used. The column temperature is 28°C, and the mobile phase is 1% formic acid water (A)-acetonitrile (B) solution, program elution (see Table 1). The volume flow is 0.3 mL min^−1^, and the injection volume is 2 *μ*L (Figure 1).

#### 3.2.4. Mass Spectrometric Conditions

Ionization method: electrospray ionization (ESI); ion polarity: negative ion (negative); detection mode: selective ion monitoring (SIM); cleavage voltage: Timosaponin AI, 60 V; Anemarrhenasaponin Ia, 82 V; Anemarrhenasaponin AII, 78 V; Timosaponin AIII, 380 V; Timosaponin BII, 88 V; Timosaponin BIII, 90 V; Anemarrhenasaponin I, 78 V; and Mangiferin, 50 V. Quantitative analysis of the mass-to-charge ratio (m/z): Timosaponin AI, 577.22; Anemarrhenasaponin AII, 755.29; Timosaponin AIII, 739.48; Timosaponin BII, 919.41; Timosaponin BIII, 901.61; Anemarrhenasaponin I, 757.35; Anemarrhenasaponin Ia, 771.35; and Mangiferin, 421.03; dry gas volume flow rate, 800 L/h; dry gas temperature, 400°C; capillary voltage, 2500 V; atomizer pressure, 24.35 kpa (35psi).

#### 3.2.5. Content Determination

Take three samples of raw and salt Anemarrhenae Rhizoma in parallel, prepare the test solution according to Section 3.2.1, detect according to the conditions under Sections 3.2.3 and 3.2.4, process the data with MassLynx V4.1, and detect the contents of 8 components in raw and salt Anemarrhenae Rhizoma.

### 3.3. Methodological Investigation

#### 3.3.1. Linear Relationship, LOD, and LOQ

8 kinds of reference substances were injected into the LC/MS chromatograph, and the peak area (Y) was used for linear regression of the analyte injection mass concentration (X). The signal-to-noise ratio (S/N) ≥10 was the LOQ of the above compounds, and S/N ≥ 3 is the LOD of the above compounds. The results of linear range, regression equation, correlation coefficient, LOD, and LOQ are shown in Table 2. The results show that the 8 components are within their respective linear ranges, *r* > 0.9990, and the linear relationship is good.

The article "Study on the Effects of Chinese Materia Medica Processing on the Hypoglycemic Activity and Chemical Composition of Anemarrhenae Rhizoma" was published in 2021. Journal: Evid Based Complement Alternat Med.

#### 3.3.2. Precision Test

Take a mixed reference solution with a known concentration, inject 6 consecutive samples under the conditions of Section 3.2, and calculate peak area. The RSD of the peak areas of Timosaponin AI, Anemarrhenasaponin AII, Timosaponin AIII, Timosaponin BII, Timosaponin BIII, Anemarrhenasaponin I, Anemarrhenasaponin Ia, and Mangiferin are 1.21%, 1.54%, 1.11%, 1.36%, 1.52%, 1.25%, 1.84%, and 1.59%, respectively, indicating that the precision of the instrument is good.

#### 3.3.3. Stability Test

Take the same samples' solution (raw Anemarrhenae Rhizoma powder) and analyze at 0, 2, 4, 6, 8, 12, and 24 hours under the condition of Section 3.2 to determine the peak areas of Timosaponin AI, Anemarrhenasaponin AII, Timosaponin AIII, Timosaponin BII, Timosaponin BIII, Anemarrhenasaponin I, Anemarrhenasaponin Ia, and Mangiferin. The RSD values of them were 1.53%, 1.56%, 1.97%, 1.51%, 1.66%, 1.45%, 1.74%, and 1.49%, respectively, indicating that the solution was stable within 24 hours.

#### 3.3.4. Repetitive Test

Take 6 samples of the same batch of powder, prepare the test product according to the method under Section 3.1, and analyze the samples under the conditions under Section 3.2 to calculate the contents of 8 components. The results show that Timosaponin AI, Anemarrhenasaponin AII, Timosaponin AIII, Timosaponin BII, Timosaponin BIII, Anemarrhenasaponin I, Anemarrhenasaponin Ia, and Mangiferin RSD were 1.70%, 1.93%, 1.72%, 1.49%, 1.94%, 1.67%, 1.84%, and 1.37%, respectively, indicating that the method has good repeatability.

#### 3.3.5. Sampling Recovery Test

Accurately weigh 0.1 g of raw Anemarrhenae Rhizoma powder (Timosaponin AI, 0.401%; Anemarrhenasaponin AII, 0.264%; Timosaponin AIII, 1.286%; Timosaponin BII, 3.544%; Timosaponin BIII, 2.179%; Anemarrhenasaponin I, 1.450%; Anemarrhenasaponin Ia, 0.982%; Mangiferin, 3.365%) in parallel 6 copies, accurately add the above 8 components of the reference substance stock solution in an appropriate amount, respectively, prepare the test solution and measure, and then calculate the recovery rate. It is calculated that the average recovery rates of the sample addition of Timosaponin AI, Anemarrhenasaponin AII, Timosaponin AIII, Timosaponin BII, Timosaponin BIII, Anemarrhenasaponin I, Anemarrhenasaponin Ia, and Mangiferin are, respectively, 98.88%, 98.77%, 99.51%, 99.69%, 99.26%, 100.69%, 99.37%, and 99.47%, and the RSD were 1.57%, 1.82%, 0.93%, 0.90%, 1.26%, 1.01%, 1.26%, and 2.01%.

The article "Study on the Effects of Chinese Materia Medica Processing on the Hypoglycemic Activity and Chemical Composition of Anemarrhenae Rhizoma" was published in 2021. Journal: Evid Based Complement Alternat Med.

## 4. Experimental Results

### 4.1. Effects of AR and SAR on Fasting Plasma Glucose (FBG) in Type 2 Diabetic db/db Mice

Compared with the db/db control group, the fasting blood glucose values of the mice in each administration group decreased (*p* < 0.01 or *p* < 0.05) after 7 days of administration. After 14 days, the fasting blood glucose values of mice in the group of AR and SAR with ethanol extract were significantly reduced (*p* < 0.01). It shows that Anemarrhenae Rhizoma can improve the fasting blood glucose level of db/db mice and has the effect of glucose-lowering. The ethanol extract of SAR has a better effect. The results are shown in Table 3 and Figure 2.

### 4.2. Effects of AR and SAR on Glucose Tolerance (OGTT) in Type 2 Diabetic db/db Mice

Compared with the db/db control group, after glucose load, the ethanol extract of SAR group significantly decreased blood sugar and glucose tolerance (AUC means glucose tolerance) at 0.5, 1, and 2 h (*p* < 0.01), while after 1 h and 2 h, the blood sugar and glucose tolerance of the water decoction group of AR and SAR and the ethanol extract group of SAR were significantly reduced (*p* < 0.01), indicating that Anemarrhenae Rhizoma has a good effect on improving glucose tolerance. The ethanol extract of SAR has the best effect. The results are shown in Table 4 and Figure 3.

### 4.3. Effects of AR and SAR on HbAlc, RESISTEIN, and FINS of Type 2 Diabetic db/db Mice

Compared with the db/db control group, the water decoction and ethanol extract of AR and SAR had significant improvement on HbAlc, FINS, HOMA-IR, ISI, and RESISTEIN (*p* < 0.01 or *p* < 0.05), and the ethanol extract of SAR was superior to the water decoction. It indicated that the effect of improving insulin resistance of ESAR is the best. The results are shown in Table 5 and Figure 4.

### 4.4. Effects of AR and SAR on SOD, MDA, and NO in Type 2 Diabetic db/db Mice

Compared with the db/db control group, the ethanol extract of SAR could significantly improve the effects of superoxide dismutase (SOD) and nitric oxide (NO) in the pancreas of type 2 diabetic mice (*p* < 0.01). The water decoction of AR and SAR and the ethanol extract of AR could also increase the content of nitric oxide (NO) in the pancreas of diabetic mice (*p* < 0.05). The ethanol extract of SAR has the best curative effect. The results are shown in Table 6 and Figure 5.

### 4.5. Measurement Results of 8 Components of the Sample

According to calculations, the contents of these 8 components in the ethanol extract of AR and SAR are higher than those in the water decoction, and the contents of the ethanol extract of SAR are the highest, which proves that the hypoglycemic effect of SAR is better than that of AR. The results are shown in Table 7 and Figure 6.

The article "Study on the Effects of Chinese Materia Medica Processing on the Hypoglycemic Activity and Chemical Composition of Anemarrhenae Rhizoma" was published in 2021. Journal: Evid Based Complement Alternat Med.

## 5. Discussion and Conclusions

This paper focuses on the hypoglycemic effects of AR, which is enhanced after being stir-baked with salt water, as reported in our previous research.

In view of the fact that oxidative stress [19] is the main cause of aggravated impairment and dysfunction of pancreatic *β*-cells [20] in recent studies of type 2 diabetes mellitus, in addition to the basic indicators, such as fasting blood sugar, serum insulin, and glucose tolerance, SOD, NO, and MDA were also detected, which can reflect oxidative stress. Especially in the pathogenesis of type 2 diabetes mellitus, oxidative stress as the central link of pancreatic *β*-cell damage is more obvious. Oxidative stress can block insulin action pathways leading to insulin resistance (IR), reduce the insulin gene expression, and promote *β*-cell apoptosis [21]. In scientific research, the levels of oxidative stress are mainly determined by reactive oxygen species (ROS) [22], reactive nitrogen species (RNS) [23], and lipid peroxides. ROS induces oxidative stress *in vivo*, but it is difficult to determine directly because of its instability. RNS mainly includes nitric oxide and peroxynitrite anion. Lipid peroxide is the product of unsaturated fatty acid by ROS, which can indirectly reflect the level of oxidative stress *in vivo*. MDA is commonly used as product index, and SOD plays an increasingly important role in the body's antioxidant mechanism as antioxidant enzyme, which cannot be ignored.

Anemarrhenae Rhizoma stir-baked with salt water can significantly improve the activity of pancreatic islet *β*-cells, reduce the content of NO in cells, and can significantly increase the activity of SOD in pancreatic *β*-cells, as well as reduce MDA activity [7]. The mechanism of its damage to pancreatic *β*-cells may be related to the enhancement of cells' ability to scavenge oxygen free radicals, resistance to exogenous NO, inhibition of MDA factor, and effective protection of pancreatic *β*-cells.

The research results have shown that compared with the water decoction, the contents of Timosaponin AI, Anemarrhenasaponin AII, Timosaponin AIII, Timosaponin BII, Timosaponin BIII, Anemarrhenasaponin I, Anemarrhenasaponin Ia, and Mangiferin in the ethanol extract of AR and SAR were increased, and the 8 components both in the water decoction and in the ethanol extract of SAR were higher than those of AR.

The research results also suggest that SAR has an improved therapeutic effect on carbohydrate metabolism and islet damage in diabetic mice. SAR is better than AR, and the ethanol extract of SAR has the most significant effect. Its hypoglycemic mechanism is related to reducing fasting blood glucose, improving glucose tolerance and insulin resistance, and protecting and repairing pancreatic islet tissue. It also suggests that these saponins are the material basis for the hypoglycemic effect of SAR. The hypoglycemic effect of the ethanol extract of SAR is better than that of the water decoction. The reason maybe the increase of the content of Timosaponin AIII, Timosaponin BIII, Mangiferin, and other components in the ethanol extract of SAR, which strengthens the hypoglycemic effect of SAR.

The article "Study on the Effects of Chinese Materia Medica Processing on the Hypoglycemic Activity and Chemical Composition of Anemarrhenae Rhizoma" was published in 2021. Journal: Evid Based Complement Alternat Med.

Anemarrhenae Rhizoma stir-baked with salt water has a long history of application, but the research on how processing enhances its hypoglycemic effect is very limited. The hypoglycemic effect experiment was combined with the analysis of chemical components to explain the influence of processing on the hypoglycemic effect of Anemarrhenae Rhizoma, which explains the traditional theory of processing in enhancing the effect of Anemarrhenae Rhizoma to nourish Yin for lowering fire from a modern point of view. It not only proves that the use of SAR in the treatment of diabetes conforms to the traditional Chinese medicine theory but also uses modern scientific knowledge to explain the traditional Chinese medicine theories, which can provide a useful modern research basis for the clinical use of SAR.

## Figures and Tables

**Figure 1:** Total ion chromatography of reference substances (a), ethanol extract from Anemarrhenae Rhizoma (b), ethanol extract from salt Anemarrhenae Rhizoma (c), water decoction from Anemarrhenae Rhizoma (d), and water decoction from salt Anemarrhenae Rhizoma (e) (1: Mangiferin; 2: Timosaponin BII; 3: Timosaponin BIII; 4: Anemarrhenasaponin I; 5: Anemarrhenasaponin AII; 6: Anemarrhenasaponin Ia; 7: Timosaponin AIII; 8: Timosaponin AI).

**Figure 2:** The fasting blood glucose (FBG) of mice in WAR, WSAR, EAR, and ESAR groups on the 0, 7, and 14 days after administration; ^*∗*^*p* < 0.05 and ^*∗∗*^*p* < 0.01 vs. control group.

**Figure 3:** The blood sugar and glucose tolerance (AUC) of mice in WAR, WSAR, EAR, and ESAR groups on the 0, 0.5, 1, and 2 h after administration; ^*∗*^*p* < 0.05 and ^*∗∗*^*p* < 0.01 vs. control group.

**Figure 4:** The HbAlc, FINS, HOMA-IR, ISI, and RESISTEIN of mice in WAR, WSAR, EAR, and ESAR groups after administration; ^*∗*^*p* < 0.05 and ^*∗∗*^*p* < 0.01 vs. control group.

**Figure 5:** The SOD, MDA, and NO of mice in WAR, WSAR, EAR, and ESAR groups after administration; ^*∗*^*p* < 0.05 and ^*∗∗*^*p* < 0.01 vs. control group.

**Figure 6:** Mass fraction of 8 components in different extracts of AR and SAR in EAR, ESAR, WAR, and WSAR groups.

The article "Study on the Effects of Chinese Materia Medica Processing on the Hypoglycemic Activity and Chemical Composition of Anemarrhenae Rhizoma" was published in 2021. Journal: Evid Based Complement Alternat Med.

**Table 1:** Mobile phase elution conditions.

Time (min)	Acetonitrile (%)	Water (%)
0.0	10	90
1.0	20	80
2.0	22	78
2.5	30	70
5.5	30	70
6.0	40	60
7.5	42	58
10.5	60	40
12	80	20
12.1	10	90
13.0	10	90

**Table 2:** Regression equations, linear ranges, correlation coefficients, LOD, and LOQ of 8 compounds.

Component	Regression equation	*r*	Linear range (*μ*g·ml^−1^)	LOD (ng·ml^−1^)	LOQ (ng·ml^−1^)
Anemarrhenasaponin AI	*Y* = 36672.5*X*+31.8912	0.9992	0.174–3.383	0.82	9.29
Anemarrhenasaponin AII	*Y* = 58521*X*+17833	0.9998	0.438–3.672	1.85	7.22
Anemarrhenasaponin AIII	*Y* = 272256*X*+12157.5	0.9998	1.821–5.539	0.81	6.96
Anemarrhena saponin BII	*Y* = 435408*X*+1514.71	0.9995	0.845–5.230	4.51	15.48
Anemarrhenasaponin BIII	*Y* = 315345*X*+359.815	0.9992	0.904–5.087	2.53	8.42
Anemarrhenasaponin I	*Y* = 841050*X*+22285.6	0.9997	0.905–4.782	3.28	12.37
Anemarrhenasaponin Ia	*Y* = 1846.99*X*+21.472	0.9999	0.806–4.385	2.74	10.31
Mangiferin	*Y* = 9082.41*X*+4205.51	0.9998	1.073–5.983	0.81	2.31

**Table 3:** The effect of different extracts of AR and SAR on FBG in diabetic mice ($\bar{x}$ ± s, *n* = 6).

Group	Dosage (g·kg^−1^)	FBG (mmol·L^−1^)		
		Preadministration	7 d after administration	14 d after administration
db/m normal control group	―	3.73 ± 0.42^*∗∗*^	3.20 ± 0.75^*∗∗*^	3.75 ± 0.37^*∗∗*^
db/db control group	―	20.05 ± 0.33	20.13 ± 0.25	19.87 ± 0.61
WAR	2.5	20.34 ± 2.05	17.91 ± 1.55^*∗*^	12.03 ± 1.39^*∗*^
WSAR	2.5	20.40 ± 2.22	16.11 ± 1.12^*∗*^	10.27 ± 1.43^*∗*^
EAR	2.5	20.88 ± 1.45	14.79 ± 2.28^*∗∗*^	6.98 ± 0.89^*∗∗*^
ESAR	2.5	20.62 ± 1.95	13.74 ± 1.98^*∗∗*^	5.82 ± 0.71^*∗∗*^

Compared with the db/db control group, ^*∗*^*p* < 0.05 and ^*∗∗*^*p* < 0.01.

**Table 4:** Effects of different extracts of AR and SAR on OGTT in diabetic mice ($\bar{x}$ ± s, *n* = 6).

Group	Dosage (g·kg^−1^)	0 h (mmol·L^−1^)	0.5 h (mmol·L^−1^)	1 h (mmol·L^−1^)	2 h (mmol·L^−1^)	AUC (mmol·L^−1^)
db/m normal control group	―	3.24 ± 0.27^*∗∗*^	11.32 ± 0.45^*∗∗*^	8.71 ± 2.07^*∗∗*^	5.14 ± 1.32^*∗∗*^	18.34 ± 3.45^*∗∗*^
db/db control group	―	18.05 ± 0.27	29.97 ± 1.06	25.02 ± 3.05	20.02 ± 2.07	57.89 ± 3.98
WAR	2.5	12.07 ± 1.35^*∗*^	21.12 ± 0.35^*∗*^	14.11 ± 1.52^*∗*^	10.17 ± 0.83^*∗∗*^	35.69 ± 5.92^*∗*^
WSAR	2.5	11.07 ± 1.23^*∗*^	20.12 ± 0.50^*∗*^	12.86 ± 1.48^*∗*^	9.34 ± 0.71^*∗∗*^	32.45 ± 5.07^*∗∗*^
EAR	2.5	10.84 ± 0.96^*∗*^	18.87 ± 2.81^*∗*^	12.74 ± 0.82^*∗*^	8.18 ± 1.96^*∗∗*^	27.66 ± 4.98^*∗∗*^
ESAR	2.5	5.84 ± 0.56^*∗∗*^	14.11 ± 2.38^*∗∗*^	11.37 ± 0.59^*∗∗*^	6.35 ± 1.76^*∗∗*^	24.87 ± 4.16^*∗∗*^

Compared with the db/db control group, ^*∗*^*p* < 0.05 and ^*∗∗*^*p* < 0.01.

**Table 5:** Effects of different extracts of AR and SAR on HbAlc, RESISTEIN, and FINS in type 2 diabetic db/db mice ($\bar{x}$ ± s, *n* = 6).

Group	Dosage (g·kg^−1^)	HbAlc (mmol·L^−1^)	FINS (mU·L^−1^)	HOMA-IR	ISI	RESISTEIN (pg·mL^−1^)
db/m normal control group	―	9.87 ± 0.84^*∗∗*^	10.84 ± 0.42^*∗∗*^	1.89 ± 0.33^*∗∗*^	−3.86 ± 0.08^*∗∗*^	125.3 ± 3.37^*∗∗*^
db/db control group	―	16.67 ± 2.24	20.11 ± 3.01	17.76 ± 2.54	−5.99 ± 0.14	160.2 ± 8.23
WAR	2.5	12.07 ± 1.48^*∗*^	17.05 ± 2.60^*∗*^	11.84 ± 1.90^*∗*^	−5.42 ± 0.38	148.9 ± 5.99^*∗*^
WSAR	2.5	9.68 ± 0.34^*∗∗*^	16.23 ± 2.44^*∗*^	10.12 ± 1.84^*∗*^	−5.32 ± 0.35	145.1 ± 5.34^*∗*^
EAR	2.5	9.38 ± 2.66^*∗∗*^	15.78 ± 1.80^*∗*^	7.49 ± 1.88^*∗∗*^	−4.92 ± 0.27^*∗*^	139.3 ± 6.61^*∗*^
ESAR	2.5	9.31 ± 3.06^*∗∗*^	14.42 ± 1.37^*∗∗*^	6.13 ± 1.03^*∗∗*^	−4.42 ± 0.29^*∗*^	131.1 ± 5.12^*∗∗*^

Compared with the db/db control group, ^*∗*^*p* < 0.05 and ^*∗∗*^*p* < 0.01.

The article "Study on the Effects of Chinese Materia Medica Processing on the Hypoglycemic Activity and Chemical Composition of Anemarrhenae Rhizoma" was published in 2021. Journal: Evid Based Complement Alternat Med.

**Table 6:** Effects of different extracts of AR and SAR on SOD, MDA, and NO in type 2 diabetic db/db mice ($\bar{x}$ ± s, *n* = 6).

Group	Dosage (g·kg^−1^)	SOD (ng·mL^−1^)	MDA (nmol·mL^−1^)	NO (*μ*mol·mL^−1^)
db/m normal control group	―	7.22 ± 0.18^*∗∗*^	1.93 ± 0.63^*∗∗*^	14.03 ± 2.15^*∗∗*^
db/db control group	―	4.15 ± 0.33	6.45 ± 0.49	50.05 ± 7.84
WAR	2.5	4.02 ± 0.76	6.95 ± 0.48	29.06 ± 8.56^*∗*^
WSAR	2.5	4.29 ± 0.82	6.07 ± 0.41	27.67 ± 8.12^*∗*^
EAR	2.5	5.15 ± 0.37^*∗∗*^	5.18 ± 0.80	22.93 ± 4.27^*∗∗*^
ESAR	2.5	5.95 ± 0.31^*∗∗*^	4.33 ± 0.73	18.49 ± 3.71^*∗∗*^

Compared with the db/db control group, ^*∗*^*p* < 0.05 and ^*∗∗*^*p* < 0.01.

**Table 7:** Mass fraction of 8 components in different extracts of AR and SAR.

Group	Mass fraction (mg·g^−1^)							
	Anemarrhenasaponin AI	Anemarrhenasaponin AII	Anemarrhenasaponin AIII	Anemarrhenasaponin BII	Anemarrhenasaponin BIII	Anemarrhenasaponin I	Anemarrhenasaponin Ia	Mangiferin
EAR	0.401	0.264	1.286	3.544	2.179	1.450	0.982	3.365
ESAR	0.427	0.271	1.949	4.918	2.742	1.859	1.203	4.174
WAR	0.326	0.247	0.932	3.355	1.822	0.956	0.709	2.987
WSAR	0.349	0.280	1.429	4.261	2.427	1.367	1.161	3.292

## Data Availability

The data used to support the findings of this study are available from the corresponding author upon request.

## Abbreviations

AR: Anemarrhenae Rhizoma
SAR: Anemarrhenae Rhizoma stir-baked with salt water
EAR: Ethanol extract from Anemarrhenae Rhizoma
ESAR: Ethanol extract from Anemarrhenae Rhizoma stir-baked with salt water
WAR: Water decoction from Anemarrhenae Rhizoma
WSAR: Water decoction from Anemarrhenae Rhizoma stir-baked with salt water
FBG: Fasting blood glucose
OGTT: Oral glucose tolerance test
HbA1c: Glycated hemoglobin
RESISTEIN: Serum resistin
FINS: Fasting insulin
SOD: Superoxide dismutase
MDA: Malondialdehyde
NO: Nitric oxide.
